# Evaluation of the Effect of Four Bioactive Compounds in Combination with Chemical Product against Two Spider Mites *Tetranychus urticae* and *Eutetranychus orientalis*(Acari: Tetranychidae)

**DOI:** 10.1155/2022/2004623

**Published:** 2022-08-22

**Authors:** Amine Assouguem, Mohammed Kara, Amal Ramzi, Saoussan Annemer, Alicja Kowalczyk, Essam A. Ali, Bushra Abdulkarim Moharram, Abderrahim Lazraq, Abdellah Farah

**Affiliations:** ^1^Laboratory of Applied Organic Chemistry, Faculty of Sciences and Technologies, Sidi Mohamed Ben Abdellah University, Route d'Imozzer, Fez, Morocco; ^2^Laboratory of Functional Ecology and Environment, Faculty of Sciences and Technology, Sidi Mohamed Ben Abdellah University, Imouzzer Street, P.O. Box 2202, Fez, Morocco; ^3^Laboratory of Biotechnology, Conservation and Valorization of Natural Resources (LBCVNR), Faculty of Sciences Dhar EI Mehraz, Sidi Mohamed Ben Abdellah University, B. P. 1796, Fez 30000, Morocco; ^4^Department of Environmental Hygiene and Animal Welfare, Wrocław University of Environmental and Life Sciences, Chełmo ´nskiego 38C, Wrocław 51-630, Poland; ^5^Department of Pharmaceutical Chemistry, College of Pharmacy, King Saud University, Riyadh 11451, Saudi Arabia; ^6^Department of Pharmacognosy, Faculty of Pharmacy, Sanaa University, Sanaa, Yemen

## Abstract

Currently, pests control using chemical acaricides constitutes worries for ecologists and health care people as these chemical products create damage to the ecosystem as well as the development of spider mites resistance. Such concerns request deep and rapid feedback by looking for new alternative and eco-friendly methods. In recent years, a new field is evolving in the use of essential oils in pest management practices. Essential oils have been considered as potential pest management agents, because they demonstrate to have a broad range of bioactivity, possess contact, and fumigant toxicity. In addition, the major advantages of many plant-based acaricides lie in their low toxicity to agroecosystems. Botanical acaricides composed of essential oils may prove to be a good choice for the more persistent synthetic acaricides. In this study, the acaricidal effect of four plant-derived essential oils against adults of the two important crop pests, *Tetranychus urticae* (Koch) 1836 and *Eutetranychus orientalis* (Klein) 1936 are studied. The fumigant toxicity revealed that all the essential oils tested *Mentha pulegium* L., *Lavandula stoechas* L., *Rosmarinus officinalis* L., and *Origanum compactum* Benth (Lamiaceae family) displayed an acaricidal effect. At the highest dose (625 µl/ml), mortalities recorded were found between 91 and 98% and 92 and 99% at 24 and 48 h, respectively, for *T. urticae*, and between 90 and 98% and 94 and 99% at 24 and 48 h, respectively, for *E. orientalis*. The *M. pulegium* L. essential oil represents the highest activity against *E. orientalis* and *T. urticae*. For the binary combination between the EOs (essential oils) and the acaricide based on the active ingredient acequinocyl, the results showed that the mixture of *O. compactum* EO (essential oil) + acequinocyl exhibited an important acaricidal effect on *T. urticae* and *E. orientalis* with 99% at 24 h and 100% at 48 h of mortality, followed by *M. pulegium* EO + acequinocyl with 92% at 24 h and 95% at 48 h for *T. urticae* as well as 99% at 24 h and 100% at 48 h for *E. orientalis* of mortality. Whereas, the mixture of *L. stoechas* EO + acequinocyl presented the lowest activity against *T. urticae* and *E. orientalis* with 82–87% at 24 h and 86–90% at 48 h, respectively. The mixtures (*M. pulegium* EO + acequinocyl, *R. officinalis* EO + acequinocyl, and *O. compactum* EO + acequinocyl) exerted a high acaricidal effect against *E. orientalis*. These promising results could help to develop botanical pesticides that could be used in integrated pest management.

## 1. Introduction

Spider mites including *Tetranychus urticae* (Koch) 1836 and *Eutetranychus orientalis* (Klein) 1936 are a major pest of citrus in many countries including Morocco [1, 2]. These two pests cause considerable losses to citrus crops [3, 4]. In recent years, these pests have become of great economic importance [5, 6], by sucking the cellular juice of the leaves causing yellowing, necrosis, and leaf fall which weakens the plant and reduces the photosynthetic capacity [7]. Their control is often provided by intensive and preventive chemical control [8, 9]. In Morocco, the Acequinocyl, Abamectin, Malathion, Spirodiclofen, Bifenazate, Fenpyroximate, Fenazaquin, Tebufenpyrad, Propargite, Milbemectine, Bifenthrine, Dicofol, Clofentezine, Maltodextrine, and Pyridaben are the most acaricides employed to control spider mites including *T. urticae* and *E. orientalis* under greenhouses and field [1,10]. Despite advantages such as easy use, the decrease of pests numbers, and their immediate action when compared with natural extracts from plants [11]. This approach has considerable limitations; the examination of the spectrum activity of the functional components used throughout the globe demonstrates that 72% of insecticides, 28% of fungicides, and 46% of acaricides are globally toxic toward auxiliary arthropods and public health [12, 13].

Acequinocyl is a naphthoquinone compound discovered in the 1970s by DuPont [14]. It is a proacaricide that breaks down into the active metabolite, a deacetylated product. A mechanistic study showed that the deacetylated metabolite of acequinocyl inhibits respiration in mitochondria at the ubiquinol oxidation site (Q0) of complex III of the electron transfer chain [15, 16].

The control by *Mentha pulegium, Lavandula stoechas, Rosmarinus officinalis*, and *Origanum compactum* (Lamiaceae family) can be used as alternative approaches for control. Essential oils include a plentiful interest for researchers who always try through their scientific studies to discover the great potential of these substances as anti-inflammatory, antioxidant, antimicrobial, and AC agents [17, 18]. Plants from the Lamiaceae family including *M. pulegium*, *L. stoechas*, *R. officinalis*, and *O. compactum* are well known for their acaricidal dynamic biological activities and many reports have demonstrated the existence of different compounds like terpenes, iridoids, flavonoids, and phenolic constituents the species of this family [19, 20]. Moreover, it had been conveyed that the two Lamiaceae plants, *M. pulegium* and *R. officinalis* have multiple significant acaricidal activities against spider mites [21, 22]. *M. pulegium* possesses several acaricidal properties; this aromatic plant has demonstrated antioxidant and anticholinesterase, anthelmintic, antimicrobial, insecticidal, and acaricidal effects [23–25]. Similarly, *R. officinalis* is well known for its beneficial effect as a medicinal mechanism and it also showed an acaricidal potential against pests [26]. The objective of this work was to evaluate the acaricidal effect of four essential oils derived from *M. pulegium, L. stoechas, R. officinalis*, and *O. compactum*, alone and in combination with a chemical acaricide based on acequinocyl, against two spider mites, *T. urticae* and *E. orientalis.*

## 2. Materials and Methods

### 2.1. Plant Material and Extraction of Essential Oils

Samples of *Lavandula stoechas, Mentha pulegium, and Origanum compactum* (Lamiaceae family) were collected between April and June (the flowering stage) in the mountainous area that is located in the rural community of Timezgana (Northeastern Morocco, 34°34′48″ North, 4°43′48″ West), at an altitude of approximately 800 m.

Samples of *R. officinalis* come from the experimental garden of the Faculty of Science and Technology of Fez. The collected plants were identified at the National Agency for Medicinal and Aromatic Plants in Taounate, Morocco.

These products were chosen on the basis of their availability and their effectiveness as a natural acaricide.

### 2.2. Chromatographic Analysis

Chemical analysis of all essential oils was realized using gas chromatography coupled with mass spectrometry (GC/MS) and coupled with flame ionization detection (GC-FID). The GC/MS analysis was utilized for identification, while GC-FID analysis was used for the quantification of components.

#### 2.2.1. Gas Chromatography (GC-FID) Analysis

Gas chromatography analyses for all the samples were realized using a Hewlett-Packard (HP 6890) gas chromatograph equipped with an HP-5 capillary column (30 m × 0.25 mm, film thickness of 0.25 *µ*m), FID a detector, and an injector fixed at 275°C. The oven temperature was at 50°C for 5 min and then increased to 250°C at 4°C/min. The nitrogen (1.8 ml/min) was utilized as carrier gas. The samples were diluted to 1/50 in methanol and the injected volume was 1 *µ*l using a split mode ratio: 1/50, flow: 72.1 ml/min. The relative proportions of the EOs components were reported as percentages determined using peak-area normalization. The retention indices (RI) on HP-5 MS column, were identified using homologous series of (C8–C28) alkanes.

#### 2.2.2. GC/MS Analysis

Chemical analysis was carried out using a Hewlett-Packard gas chromatograph (HP 6890) coupled with a mass spectrometer (HP 5973). The column utilized was HP-5MS (cross-linked 5% PHME siloxane; 30 m × 0.25 mm, film thickness 0.25 *µ*m). The column temperature was set at 50°C and increased to 250°C at a rate of 2°C/min. The carrier gas is helium at 1.5 ml/min, using a split mode ratio: 1/74.7, flow rate: 112 ml/min. MS identities of components were confirmed using the NIST 98 spectral library. The ion source temperature of 230°C with ionization voltages of 70 eV and a scan mass range of 35–450 m/z. The identification of the components was also confirmed by comparing the elution order of the compounds with the relative retention indices reported in the literature.

### 2.3. Spider Mites

The adult spider mites of *T. urticae* and *E. orientalis* (Acarina: Tetranychidae) were collected from a farmer in Fez city 34°02′36″N, 05°00′12″W planted by (*Citrus aurantium* L., 1753) not previously treated with chemical products (Acaricides). The collected leaves were transferred directly into referenced polyethylene bags to the laboratory for inspection. *T. urticae* and *E. orientalis* spider mites on each leaf were determined and counted on both leaf surfaces using a binocular microscope before and after the addition of the tested products.

### 2.4. Toxicity Test

The acaricidal tests were conducted according to the methodology of Sertkaya et al. (2010) with slight modifications. Firstly, various doses (39.06, 78.125, 156.25, 312.5, and 625 *µ*l/L) of each EO and the chemical acaricide (Kanemite, 15%) were prepared. Thereafter, 20 adults of each *Tetranychidae* species (*T. urticae* and *E. orientalis*) survived in citrus leaves were placed in glass petri dishes (90 mm × 20 mm). Disks of filter papers that were previously attached to the interior surface of the petri dish cover were impregnated with 10 *µ*l of each concentration. DMSO (0.01%) was used as a negative control. Five replications of treatments and controls were carried out. The toxicity was evaluated after 24 and 48 h of exposure, and the mortality was calculated using the formula of Abbott (1)

(1) $$\begin{array}{c} \%\text{Mortality Corrected}=\left[\frac{\%\text{Mortality Observed}-\%\text{Mortality Control}}{100-\%\text{Mortality Control}}\right]\times 100. \end{array}$$

### 2.5. Statistical Treatment

Mortality percentages were analyzed by the SPSS software (IBM SPSS Statistics 25.0). The obtained results were also examined with OriginPro 2021 software to determine the significant effect between mean values using the Tukey test (a probability of *p* ≤ 0.05 is regarded as statistically significant). The different principal component analysis was carried out by using the JMP Pro 14. The LD_50_ values were estimated using a probit regression analysis (with SPSS software) according to Finney's mathematical methods [27].

## 3. Results

### 3.1. Chemical Composition of the Four Tested EOs

As presented in Table 1, *M. pulegium* EO was dominated by *r* (+)-pulegone (74.03%), carvone (5.45%), and dihydrocarvone (3.66%). *L. stoechas* EO was characterized by camphor (43.97%), fenchone (30.39%), camphene (4.09%), borneol (2.92%), and *α*-pinene (2.84%); whereas 1,8 cineole (29.31%), camphor (24,66%), and *α*-pinene (12.76%) were the main components in *R. officinalis*. EO. Thymol (30.05%), carvacrol (25.33%), and *γ*-Terpinene (17.23%) presented the main volatile components in *O. compactum* EO.

### 3.2. Toxicity of EOs on *T. urticae* and *E. orientalis*

Figures 1 and 2 illustrate the significant differences of the acaricidal effects of the four EOs and the chemical acaricide on *T. urticae* (Figure 1) and *E. orientalis* (Figure 2) according to mortality time (Figure 2(a)) and different concentration (Figure 2(b)). A significant difference (*p* < 0.05) was noted between *M. pulegium, R. officinalis, L. stoechas,* and *O. compactum* (*p*=0.008) as well as between the four EOs and acaricide (*p*=0.009) in terms of mortality (%). In addition, a significant difference was observed between concentration (C1, C2, C3, and C4) of EOs and acaricide (*p*=0.004) in terms of mortality (%). However, no significant difference (*p* > 0.05) was detected between EOs and acaricide (*p*=0.08) in terms of concentration C5, except *R. officinalis* EO for *T. urticae*. No significant difference was found between the mortality time of the four EOs and acaricide (*p*=0.18) in terms of *T. urticae* and *E. orientalis* mortality. It could be said that the mortality varies according to the oil and the acaricide tested and the treated mite species, generally; it was concentration-dependent. Indeed, *M. pulegium* and *O. compactum* EOs were the most effective against the two mites at all concentrations used, yet all EOs caused more than 90% of mortalities at the highest dose (C5: 625 µl/L). These results showed the important acaricidal potential of the different EOs. The chemical acaricide, Kanemite with the acequinocyl as the active molecule also displayed toxicity that varied in function of doses.

The lethal doses (LD_50_) values obtained for each essential oil and the chemical acaricide are presented in Table 2. It was found that *M. pulegium* EO, *O. compactum* EO, and the chemical acaricide displayed the lowest LD_50_ values on adults of *T. urticae* after 24 h (65.78, 87.92, and 36.25 µl/L air, respectively) and after 48 h of treatment (56.1, 79.72, and 32.09 µl/L air, respectively). For *E. orientalis*, the lowest LD_50_ values were obtained for *M. pulegium* EO, *R. officinalis* EO, and the acaricide after 24 h (59.10, 88.2, and 34.07 µl/L air, respectively) and after 48 h of exposure (47.37, 82.44, and 29.15 µl/L air, respectively). The Chi-square test was not significant at 5% for all samples (EOs and the acaricide), which means goodness of fit.

95% CI: 95% confidence intervals; df: degree of freedom (Total); *X*^2^: Chi-square.

### 3.3. Toxicity of the EOs and the Acaricide on *T. urticae* and *E. orientalis*

As shown in Figure 3, the four binary mixtures exhibited an important acaricidal effect on both *T. urticae and E. orientalis* after 24 and 48 h of treatment. A significant difference (*p* < 0.05) was indicated in the mortality percentage of *T. urticae* between the *M. pulegium* EO + chemical acaricide (acequinocyl), *L, stoechas* EO + chemical acaricide (acequinocyl), and *O. compactum* EO + chemical acaricide (acequinocyl; *p*=0.014), while no significant difference was identified between *M*. *pulegium* EO + chemical acaricide (acequinocyl) and *R. officinalis* EO + chemical acaricide (acequinocyl; *p*=0.031). No significant difference (*p* > 0.05) was identified between *M. pulegium* EO + chemical acaricide (acequinocyl), *R. officinalis* EO + chemical acaricide (acequinocyl), and *O. compactum* EO + chemical acaricide (acequinocyl; *p*=1.00), whereas a significant difference (*p* < 0.05) was found between *L. stoechas* EO + chemical acaricide (acequinocyl) and the three mixtures in terms of the mortality percentage of *E. orientalis* (*p*=0.544). There was no significant in the mortality time of the four EOs and acaricide in terms of *T. urticae* and *E. orientalis* (*p*=0.115). The binary combination (*M. pulegium* EO + chemical acaricide) and (*O. compactum* EO + chemical acaricide) exerted a high acaricidal effect against *T. urticae* with 92 ± 2.74–99 ± 2.23% at 24 h and 95 ± 3.54–100 ± 0.00% of mortalities, respectively. However, the mixtures (*M. pulegium* EO + chemical acaricide, *R. officinalis* EO + chemical acaricide, and *O. compactum* EO + chemical acaricide) were the most effective on spider mites adults of *E. orientalis* with 99 ± 2.24% at 24 h and 100 ± 0.00% at 48 h of mortality. These results are very relevant and proved the acaricidal potential of EOs if they compared with the individual one.

### 3.4. Principal Component Analysis

#### 3.4.1. The Effect of the Main Compounds of the Four Tested EOs and Their Acaricidal Activity

The first principal component analysis (PCA) allowed identifying the existence of correlations (positive and negative) between the major compounds of the four essential oils and the acaricidal activity against *E. orientalis* and *T. urticae* in 24 and 48 h. The correlations of the different parameters studied are shown in a correlation matrix (Table 1).

The loading plot (Figure 4(a)) and the correlation matrix (Table 3) revealed some correlation between the variables studied. A strong positive correlation (>0.7) exists between (a) *α*-pinene and LD_50_ of *T. urticae*, (b) 1,8-cineole and LD_50_ of *T. urticae*, and (c) Borneol and LD_50_ of *T. urticae*. A medium positive correlation (0.6–0.5) exists between fenchone and LD_50_ of *E. orientalis*. A strong negative correlation (>−0.7) exists between (a) dihydrocarvone and LD_50_*E. orientalis*, (b) r(+)-pulegone and LD_50_*E. orientalis*, and (c) carvone and LD_50_ of *E. orientalis*. That means that when the amount of 1,8-cineole, *α*-pinene, and borneol compounds increased with increased LD_50_ of *T. urticae*, and when the LD_50_ of *E. orientalis* was low, the amount of dihydrocarvone, r(+)-pulegone, and carvone were important. The biplot (Figure 4(b)) showed that essential oils of *L. stoechas* and *R. officinalis* are dominated by the highest amount of 1,8-cineole, *α*-pinene, borneol, and fenchone compounds and they require a high concentration to eliminate *E. orientalis*. However, *O. compactum* essential oil is presented with a high amount of thymol and *α*-terpinene compounds. The *M. pulegium* was characterized by having the highest amount of r (+)-pulegone and carvone compounds and they require lowest concentration to eliminate *E. orientalis*.

Based on the result from Figures 4(a) and 4(b), it can be concluded that *M. pulegium* essential oil exhibited the best acaricide activity of the four essential oils. In fact, this can be explained by a high amount of r(+)-pulegone and carvone compounds in *M. pulegium* essential oil (74.03 and 5.45%, respectively) compared with *L. stoechas*, *R. officinalis*, and *O. compactum* (the absence of these compounds), but the contributions of others compounds should also be noted. The effect of synergy could also be the origin of this activity.

#### 3.4.2. The Effect of the Concentrations of the Four Tested EOs and Their Acaricidal Activity

The second PCA permeated to identify the similar acaricidal activity effect of essential oil and concentration, the first principal component analysis was carried out. The individuals are represented by four essential oil samples (*M. pulegium*, *L. stoechas*, *O. compactum*, and *R. officinalis*) in five different concentrations (C1, C2, C3, C4, and C5). The variables are represented by acaricidal activity against *E. orientalis* and *T. urticae* in 24 and 48 h.

The biplot (Figure 5(a)) demonstrated that the distribution of individuals (concentration) in accordance with PC1 and PC2 shows that individuals were separated into three main groups. These results indicated that the concentration has an effect on the acaricidal activity, as previously shown by ANOVA. The first group consisted of C1 (39.06 µl/ml) and C2 (78.125 µl/ml), or the low concentration. The second group is composed of C4 (312.5 µl/ml) and C5 (625 µl/ml), or the high concentration. The third groups were C3 (156.25 µl/ml), or the medium concentration. This graph indicated that when the concentration was high, the acaricidal activity against *E. orientalis* and *T. urticae* was elevated, and when the concentration was low, the acaricidal activity against *E. orientalis* and *T. urticae* was decreased. The biplot (Figure 5(b)) showed that the acaricidal activity against *E. orientalis* and *T. urticae* improved when the *M. pulegium* essential oil was used. In contrast, the *L. stoechas* and *O. compactum* essential oils revealed a medium acaricidal activity against *T. urticae*. In addition, the *R. officinalis* showed a medium acaricidal activity against *E. orientalis*.

#### 3.4.3. The Effect of the Four Mixtures Between Acaricide and Tested EOs and Their Acaricidal Activity

The third PCA was enabled to determine the similar mixtures that have the same acaricidal activity between the four mixtures studied (*M. pulegium* EO + acaricide, *R. officinalis* EO + acaricide, *O. compactum* EO + acaricide, and *L. stoechas* EO + acaricide).

The biplot (Figure 6) illustrated that the individuals (mixtures) were divided into three main groups. The first group was the mixture of *M. pulegium* EO + acaricide and *R. officinalis* EO + acaricide. The second group was the mixture of *O. compactum* EO + acaricide. The third group was *L. stoechas* EO + acaricide. The mixture of (a) *M. pulegium* EO + acaricide and (b) *R. officinalis* EO + acaricide showed the same acaricidal activity, a medium effect against the *T. urticae* and a low effect against *E. orientalis*. This graph also indicated that the acaricidal activity has been improved with the mixture of *O. compactum* EO + acaricide (synergetic effect), while the mixture of *L. stoechas* EO + acaricide presented a low acaricidal activity against the *E. orientalis* and *T. urticae* (antagonistic effect).

### 3.5. The Hierarchical Cluster Analysis

The hierarchical cluster analysis (HCA) allowed us to better classify the studied samples (the four essential oils) according to the acaricidal activity against the *E. orientalis* and *T. urticae* (Figure 7). As a confirmation of the third PCA, the individuals were divided into three main clusters: cluster 1 (*M. pulegium* EO + acaricide and *R. officinalis* EO + acaricide) characterized by a high acaricidal activity against *T. urticae*, while it was characterized by a low acaricidal activity against the *E. orientalis*. However, cluster 2 (*O. compactum* EO + acaricide) was characterized by a high acaricidal activity against the *E. orientalis* and *T. urticae*. Cluster 3 (*L. stoechas* EO + acaricide) was featured by a low acaricidal activity against the *E. orientalis* and *T. urticae*. Both the PCA and HCA concluded that the acaricidal activity against the *E. orientalis* and *T. urticae* were significantly influenced by adding the acaricide to essential oils. A synergetic effect with *O. compactum* EO + acaricide and an antagonistic effect with *L. stoechas* EO + acaricide.

## 4. Discussion

In commercial orchards, the protection against pests is currently assured by intensive and preventive chemical products. Despite advantages such as rapid action in reducing the number of pests and their ease of use compared with natural plant extracts. [20], this strategy has many limitations; the examination of the action spectrum of the active components used throughout the world reveals that 46% of acaricides are globally toxic toward auxiliary arthropods and public health [1, 28]. The extracts of plants are remarkably rich in toxins and inhibitors and can be the source of many insecticidal and acaricidal substances exploitable in the control of pests [29, 30]. On the contrary, the problem of volatility and the high cost causes several limitations of their usage [31], The essential oils lose their force against environmental conditions. Nanoformulation is a method that may preserve the pesticide performance of plant essential oils [31, 32].

Phytochemical products are environmentally friendly, target-specificity, decreased the number of applications, higher acceptability, suitability for rural areas, low cost, biodegradable, easy preparation, and universally accepted. Botanicals are used as an alternative to synthetic acaricides and have been projected as a tool in the future for spider mites control agents, which are shown to function as highly polyphagous herbivore and primary agricultural pests in the world that provokes hard damage to crops.

In this study, *M. pulegium, L. stoechas, R. officinalis, and O. compactum* (Lamiaceae family) EOs showed an acaricidal potential toward adults of the two crop pests, *T. urticae* and *E. orientalis*. Indeed, the mortality varied according to the EO tested, the concentrations used, and the mite species.

*R. officinalis* was often effective against agricultural crop pests including tetranychid mites [22, 33]. The essential oil of *R. officinalis* and mixtures of its main constituents gave good results in the control of *T. urticae* Koch, on bean and tomato plants [34].

Thymol, a hydrophobic compound, constitutes the major monoterpene in *O. compactum*; it can penetrate the compartment membrane, which diminishes its impermeability, this mechanism stimulates the entry of other components into the cytoplasm [35, 36]. There is also evidence in the literature that thymol and eugenol have a neurotoxic effect on arthropods, with different mechanisms of action. Thymol can bind to GABA receptors located in the membrane of post-synaptic neurons and disrupt the functioning of synapses [37] under laboratory conditions. A study shows that the essential oils of *O. compactum* is often toxic against *Rhyzopertha dominica* and *Sitophilus oryzae* Linnaeus, 1763 [38]. This was confirmed in our study against *T. urticae* and *E. orientalis. O. compactum* significantly inhibited oviposition of *T. urticae;* it was also toxic to females of this pest. Inhibition of fecundity exceeding 80% [39]. The essential oil of *M. pulegium* was very toxic against the strawberry spider mite *Tetranychus turkestani* Ugarov and Nikolskii, 1937 (Acari: Tetranychidae) [19]. The same results in another study were observed on *T. urticae*, a serious pest of many agricultural crops. The phytotoxicity of *M. pulegium* was significant against this pest after 24 h [40, 41].

The statistical analysis (first PCA) permed to conclude that the acaricidal activity depends on the major compounds of the essential oils tested. A strong correlation was identified between the LD_50_, dihydrocarvone and carvone. Thus, when the quantity of dihydrocarvone and carvone increased, the acaricidal activity increased. Several studies reported that the principal compound present in the essential oils of thyme and oregano increases (thujone 65.78% and carvone 59.35%) the acaricidal activities against spider mite *Tetranychus cinnabarinus* Boisd are more important [42]. In another study, 28 monoterpenes including monoterpene hydrocarbons and oxygenated monoterpenes (camphor, 3-carene, carvone, 1,8-cineole, citronellal, *β*-citronellene, dihydrocarvone, and *α*-terpineol) of essential oils obtained from different plant species were tested against adults of *Sitophilus zeamais* Motschulsky under laboratory conditions. The results show that most of the monoterpenes with high concentrations have significantly insecticidal and acaricidal effects on the tested pests [43, 44].

The second PCA showed that *M. pulegium* was found to be more effective, followed by *O. compactum* EO and *L. stoechas*. EOs acquired from multiple plants have already been tested for their potential fumigant toward pests species (Choi et al., 2006) [42]. As an example, [45] examined the fumigant toxicity of *L. stoechas* EOs against three spider mites pests attacking stored products (*Lasioderma serricorne* Fabricius 1792, *R. dominica* Fabricius 1792, and *Tribolium castaneum* Herbst, 1797), the findings of this analysis showed that this EO had strong acaricidal properties with the high rates of mortality were obtained after 24 and 48 h of fumigation*. L. stoechas* was also tested for its acaricidal action against *Tetranychus cinnabarinus* Koch, 1836, one of the most important pests, the registered LC_50_ and LC_90_ values were in the range of 2.92 and 13.0 µg/ml, respectively [42]. Author [35] also recorded an effective acaricidal effect of *L. stoechas* against *Orgyia trigotephras* Boisduval, 1828 (Lepidoptera, Lymantriidae).

The third PCA and HCA illustrated that the activity of *O. compactum* EO has been ameliorated when it is mixed with the acaricide (synergetic effect). The *R. officinalis and M. pulegium* remain have the same activity when they were mixed with the acaricide. However, the activity of *L. stoechas* reduced when it was mixed with the acaricide (antagonistic effect). Several studies confirm that the mixture of several products often triggers an antagonistic effect or a synergistic effect and all depends on the obtained combination [39, 46, 47].

Moreover, the fumigant toxicity for EOs mixtures with the chemical acaricides revealed encouraging results where the mortality reached more than 95% for both spider mites. The search for synergistic mixtures aims to reduce the concentrations needed by increasing the biological activity against the target organism. This reduction of concentration may also result in decreased toxicological and environmental risks, and lower production cost [48, 49].

## 5. Conclusions

This scientific investigation highlighted the acaricidal effect of four essential oils against two important spider mites involved in agriculture damage. The obtained results proved the acaricidal potential of the tested oils and showed the efficacy of the binary mixtures with an acaricidal product reaching the mortality to 100%. These plant-based natural products can be applied in large field applications using low concentrations (based on the LD_50_ values) and minimizing the production cost; they since could be involved in pest management programs as a new tool that could solve pest problems reducing risks to humans and the environment. Their inclusion in an integrated pest management program can contribute greatly to the achievement of the acaricide reduction objectives set by several countries and organizations. In this context, responsible agricultural organizations should actively support the development and implementation of essential integrated pest protection programs. Further studies are needed to test the toxicity of these natural products.

## Figures and Tables

**Figure 1:** Mortality rate (%) of *Tetranychus urticae* adults (a) according to mortality time. T1: 24 h; T2: 48 h, (b) according to various concentrations. C1: 39.06 *µ*l/ml, C2: 78.125 µl/ml, C3: 156.25 *µ*l/ml; C4: 312.5 *µ*l/ml, C5: 625 *µ*l/ml. Different letters indicate significant differences according to the Tukey test.

**Figure 2:** Mortality rate (%) of *Eutetranychus orientalis* adults (a) according to mortality time. T1: 24 h; T2: 48 h, (b) according to various concentrations. C1: 39.06 µl/ml, C2: 78.125 µl/ml, C3: 156.25 µl/ml; C4: 312.5 µl/ml, C5: 625 µl/ml. Different letters indicate significant differences according to the Tukey test.

**Figure 3:** Mortality rate (%) of *Tetranychus urticae* adults according to various binary mixture of EOs and acaricide. (b) Mortality rate (%) of *Eutetranychus orientalis* adults according to various binary mixture of EOs and acaricide. Mixture 1: *M. pulegium* EO + acaricide; Mixture 2: *L. stoechas* EO + acaricide; Mixture 3: *R. officinalis* EO + acaricide; Mixture 4: *O. compactum* EO + acaricide. T1: 24 h; T2: 48 h. Different letters indicate significant differences according to the Tukey's test (*p* ≤ 0.05).

**Figure 4:** Principal component analyses of the main compounds in regards to the four essential oils. (a) Loading plot of the projection of the variables (main compounds) on the first and second principal components; (b) biplot of the projection of the variables on the individuals (the four essential oils) on the first and second principal components.

**Figure 5:** Principal component analyses of acaricidal activity against *E. orientalis* and *T. urticae* adults in regards to the four essential oils and concentrations. (a) Biplot of the projection of the variables and the individuals according to concentrations on the first and second principal components; (b) biplot of the projection of the variables and the individuals according to essential oils on the first and second principal components.

**Figure 6:** Biplot of the projection of the acaricidal activity against *T. urticae* and *E. orientalis* adults and the four mixtures on the first and second principal components.

**Figure 7:** Hierarchical cluster analysis of the four mixtures against *E. orientalis* and *T. urticae* adults.

**Table 1:** The major chemical constituents of the four EOs.

Compound	% Relative peak area					
	*RI * ^*a*^	*RI * ^*b*^	*M. pulegium*	*L. stoechas*	*R. officinalis*	*O. compactum*
*α*-pinene	939	932	0.42	2.84	12.76	2.24
Camphene	953	946	—	4.09	2.47	Tr
*α*-Terpinene	1002	1007	—	—	Tr	3.45
p-Cymene	1026	1022	—	0.32	0.09	11.22
1,8- cineole	1033	1033	—	1.42	31.15	Tr
*γ*-Terpinene	1062	1024	—	0.34	—	17.23
Fenchone	1088	1087	—	30.39	—	Tr
Camphor	1143	1146	—	43.97	26.96	0.14
Borneol	1165	1166	—	2.92	5.46	0.42
Dihydrocarvone	1194	1191	3.66	—	—	—
R (+)-pulegone	1238	1233	74.03	—	Tr	—
Carvone	1242	1239	5.45	0.12	—	Tr
Thymol	1290	1293	—	—	—	30.05
Carvacrol	1298	1291	—	—	—	25.33
Total %			83.56	86.41	78.89	90.08

**Table 2:** LD_50_ values calculated for *Tetranychus urticae* and *Eutetranychus orientalis*.

Spider mites species	Sample	LD_50_ (µl/L air, 24 h, 95% CI^*∗*^)	Slope (24 h)	Intercept (24 h)	df	*X*2	LD_50_ (µl/L air, 48 h, 95% CI)	df	*X*2	Slope (48 h)	Intercept (48 h)
*Tetranychidae urticae*	*M. pulegium*	65.78 (44.63–10110.12)	1.69 ± 0.17	1.93 ± 0.38	4	4.21	56.1 (33.8–69.5)	4	4.68	1.86 ± 0.18	1.75 ± 0.41
	*L. stoechas*	100.03 (85.88–120.12)	1.80 ± 0.24	1.41 ± 0.55	4	2.64	85.35 (65.15–115.12)	4	2.89	1.87 ± 0.27	1.38 ± 0.60
	*R. officinalis*	171.87 (163.24–184.96)	1.59 ± 0.41	1.44 ± 0.91	4	1.95	141.51 (120.39–162.10)	4	2.28	1.67 ± 0.48	1.40 ± 0.07
	*O. compactum*	87.92 (68.15–99.65)	1.29 ± 0.27	2.50 ± 0.56	4	3.92	79.72 (58.9–95.42)	4	4.10	1.79 ± 0.33	1.27 ± 0.75
	Chemical acaricide	36.25 (27.77–52.48)	1.42 ± 0.37	2.79 ± 0.83	4	4.62	32.09 (19.81–61.10)	4	4.9	1.72 ± 0.35	2.21 ± 0.78

*Eutetranychus orientalis*	*M. pulegium*	59.10 (40.5–78.9)	1.86 ± 0.15	1.71 ± 0.35	4	3.99	47.37 (39.80–63.65)	4	4.51	1.91 ± 0.19	1.80 ± 0.42
	*L. stoechas*	120.87 (101.19–146.62)	1.79 ± 0.14	1.26 ± 0.31	4	1.98	100.35 (85.98–121.72)	4	2.15	1.75 ± 0.15	1.50 ± 0.33
	*R. officinalis*	88.2 (66.6–112.24)	1.76 ± 0.28	1.57 ± 0.63	4	3.10	82.44 (70.06–109.2)	4	3.84	1.89 ± 0.24	1.43 ± 0.54
	*O. compactum*	112.77 (89.5–135.7)	2.36 ± 0.24	0.16 ± 0.54	4	2.92	96.85 (81.45–140.16)	4	3.8	2.38 ± 0.27	0.28 ± 0.61
	Chemical acaricide	34.07 (25.10–50.23)	1.49 ± 0.29	2.72 ± 0.62	4	4.49	29.15 (17.43–29.65)	4	4.95	1.47 ± 0.27	2.84 ± 0.57

**Table 3:** Correlation matrix between the main compounds of the four essential oils and LD_50_ of *E. orientalis* and *T. urticae*.

	*α*-pinene	Camphene	*α*-Terpinene	p-Cymene	1,8-Cineole	*γ*-Terpinene	Fenchone	Camphor	Borneol	Dihydrocarvone	R(+)-pulegone	Carvone	Thymol	Carvacrol	LD_50_*E. orientalis*	LD_50_ *T. urticae*
*α*-pinene	1	0.39	−0.28	−0.28	0.99	−0.28	−0.21	0.4	0.92	−0.5	−0.5	−0.51	−0.28	−0.28	0.02	0.99
Camphene	0.39	1	−0.55	−0.53	0.32	−0.53	0.81	1	0.72	−0.55	−0.55	−0.53	−0.55	−0.55	0.52	0.49
*α*-Terpinene	−0.28	−0.55	1	1	−0.35	1	−0.33	−0.54	−0.47	−0.33	−0.33	−0.34	1	1	0.42	−0.27
p-Cymene	−0.28	−0.53	1	1	−0.36	1	−0.31	−0.53	−0.46	−0.35	−0.35	−0.36	1	1	0.44	−0.27
1,8-Cineole	0.99	0.32	−0.35	−0.36	1	−0.36	−0.29	0.33	0.88	−0.35	−0.35	−0.36	−0.35	−0.35	−0.14	0.96
*γ*-Terpinene	−0.28	−0.53	1	1	−0.36	1	−0.32	−0.53	−0.47	−0.34	−0.34	−0.35	1	1	0.44	−0.27
Fenchone	−0.21	0.81	−0.33	−0.31	−0.29	−0.32	1	0.81	0.19	−0.33	−0.33	−0.31	−0.33	−0.33	0.61	−0.09
Camphor	0.4	1	−0.54	−0.53	0.33	−0.53	0.81	1	0.73	−0.55	−0.55	−0.53	−0.54	−0.54	0.52	0.5
Borneol	0.92	0.72	−0.47	−0.46	0.88	−0.47	0.19	0.73	1	−0.58	−0.58	−0.58	−0.47	−0.47	0.21	0.95
Dihydrocarvone	−0.5	−0.55	−0.33	−0.35	−0.35	−0.34	−0.33	−0.55	−0.58	1	1	1	−0.33	−0.33	−0.87	−0.59
R(+)-pulegone	−0.5	−0.55	−0.33	−0.35	−0.35	−0.34	−0.33	−0.55	−0.58	1	1	1	−0.33	−0.33	−0.87	−0.59
Carvone	−0.51	−0.53	−0.34	−0.36	−0.36	−0.35	−0.31	−0.53	−0.58	1	1	1	−0.34	−0.34	−0.86	−0.6
Thymol	−0.28	−0.55	1	1	−0.35	1	−0.33	−0.54	−0.47	−0.33	−0.33	−0.34	1	1	0.42	−0.27
Carvacrol	−0.28	−0.55	1	1	−0.35	1	−0.33	−0.54	−0.47	−0.33	−0.33	−0.34	1	1	0.42	−0.27
LD_50_ *E. orientalis*	0.02	0.52	0.42	0.44	−0.14	0.44	0.61	0.52	0.21	−0.87	−0.87	−0.86	0.42	0.42	1	0.14
LD_50_ *T. urticae*	0.99	0.49	−0.27	−0.27	0.96	−0.27	−0.09	0.5	0.95	−0.59	−0.59	−0.6	−0.27	−0.27	0.14	1

## Data Availability

All related data are included within the article.
